The article "Outcomes in Emergency Department Patients with Dyspnea versus Chest Pain: A Retrospective Consecutive Cohort Study" was published in 2022. Journal: Emerg Med Int.

# Outcomes in Emergency Department Patients with Dyspnea versus Chest Pain: A Retrospective Consecutive Cohort Study

**DOI:** 10.1155/2022/4031684

**Published:** 2022-09-16

**Authors:** Erik Jemt, Magnus Ekström, Ulf Ekelund

**Affiliations:** ^1^Department of Emergency Medicine, Skåne University Hospital, 221 00 Lund, Sweden; ^2^Department of Clinical Sciences, Division of Respiratory Medicine & Allergology, Lund University, 221 00 Lund, Sweden

## Abstract

Dyspnea and chest pain are major and important causes of contact at the emergency department (ED). Dyspnea is associated with high morbidity and mortality, but data on characteristics and outcomes compared with chest pain in the ED are limited. This was a retrospective cohort study of consecutive patients with contact causes of dyspnea or chest pain at two Swedish EDs from 2010 to 2014. Hospital admittance, ED revisits, and mortality were analyzed using multivariable regression models, adjusted for ED and markers of disease severity (age, sex, centre, Charlson comorbidity index, c-reactive protein, troponin *T,* and arrival by ambulance). 29,291 patients (mean age 58.3 years; 48.9% women) with dyspnea (*n* = 8,812) or chest pain (*n* = 20,479) were included. Dyspnea patients were older than patients with chest pain (64 vs. 56 years, *p* < 0.001) and had more comorbidity and higher average blood troponin *T* and c-reactive protein levels. Dyspnea patients also had higher hospitalization rates (48% vs. 30%; adjOR (95% CI) 2.1–2.3), including the intensive care unit (1.4% vs. 0.1%; adjOR 6.9–15.9), and more ED revisits (11% vs. 7%; adjOR 1.2–1.7) in 30 days. Dyspnea patients had five-fold increased mortality compared to those with chest pain; hazard ratio (HR) 5.1 (4.8–5.4), adjusted for markers of disease severity, the mortality was two-fold higher, HR 2.2 (2.0–2.4). Compared with chest pain patients, ED dyspnea patients are older, have more comorbidity, and have worse outcomes in terms of hospitalization, morbidity, and mortality.

## 1. Introduction

Dyspnea and chest pain are major and important causes of contact at the emergency department (ED), with dyspnea comprising 5–9% and chest pain 11–13% of total ED admissions [1–3]. The two symptoms often appear together, they can be hard to differentiate, and both can be caused by heart as well as lung disorders. For instance, approximately 50% of the patients with pulmonary embolism have chest pain [4, 5], and acute coronary syndrome manifests with dyspnea in 4–11% of cases [6–8]. In addition, cardiac and lung diseases often occur together, and one can lead to the other, e.g. when chronic obstructive pulmonary disease (COPD) causes cor pulmonale [9].

The article "Outcomes in Emergency Department Patients with Dyspnea versus Chest Pain: A Retrospective Consecutive Cohort Study" was published in 2022. Journal: Emerg Med Int.

Management of chest pain, with coronary artery disease as the major underlying pathology [3, 10], is well studied, with reliable risk-stratification tools such as the HEART-score [11] and EDACS [12]. Compared to chest pain, the causes of dyspnea are more diverse such as heart diseases, infections, and lung diseases [3, 10], and there are few guidelines and tools for managing dyspnea in the ED.

ED patients with dyspnea have been reported to have higher in-hospital mortality than those with chest pain [3, 10], and compared to patients with other contact causes, dyspnea patients have a higher triage priority [2], longer hospital stay [10], and are more often admitted to intensive care [3]. Indeed, dyspnea at the ED is an independent predictor of short survival [13]. The long-term mortality after exercise testing has been compared in dyspnea and chest pain patients [14], but our knowledge of the similarities and differences in characteristics and outcomes in these patients is otherwise limited.

The aim of this study was to evaluate characteristics and outcomes in patients presenting to the ED with dyspnea compared to chest pain.

## 2. Materials and Methods

### 2.1. Study Design and Population

This was a retrospective consecutive cohort study using the Evaluation of Unknown Predictors of Electrocardiographic Changes (EXPECT) database [15, 16]. The database includes a vast amount of clinical information from 198,850 consecutive patients aged 18 years or older who presented at five EDs in Denmark and southern Sweden during 2010–2014 and had an electrocardiogram (ECG) registered. Only the first ED contact during the period was included for each person.

### 2.2. Ethical Considerations

The present study was approved by the Regional Ethics Review Board at Lund (Dnr: 2015/78, 2016/691, 2018/705). Active patient consent was waived by the ethics review board, but individuals were informed about the study and had the opportunity to decline participation.

### 2.3. Study Sites

The present study included data from the EDs of Lund University Hospital (approximately 65,000 visitors annually) and Helsingborg General Hospital (approximately 80,000 visitors annually) during 2010–2014. Both EDs used the Rapid Emergency Triage and Treatment System (RETTS) [17] for triage during the study period, which mandates an ECG in all patients with dyspnea or chest pain as the main cause of contact. Patients with an ST-elevation myocardial infarction (STEMI) were most often identified in the prehospital setting and taken directly to the angiography suite, bypassing the ED. These patients were thus not included in the study.

### 2.4. Assessments and Definitions

From the EXPECT database, we extracted the following data: patient's age, sex, previous diagnoses, Charlson comorbidity index (CCI) [18], ED arrival and departure times, arrival by ambulance or not, admittance to in-hospital or intensive care unit (ICU), length of hospital stay, ED blood tests of high sensitivity cardiac troponin *T* (hs-cTnT), c-reactive protein (CRP), and hemoglobin (Hb), as well as ED revisits and mortality within 7, 30, and 365 days. The variable “arrival by ambulance” was only available at Lund. Sensitivity analyses without adjusting for “arrival by ambulance” yielded similar findings.

The article "Outcomes in Emergency Department Patients with Dyspnea versus Chest Pain: A Retrospective Consecutive Cohort Study" was published in 2022. Journal: Emerg Med Int.

The contact causes were defined according to RETTS [17] and were in all cases registered by an experienced triage nurse. Dyspnea was defined as shortness of breath with or without relation to effort and chest pain as pain from the thoracic area with or without relation to breathing. To prevent the overlap between the two groups and ensure that they were mutually exclusive, dyspnea patients with chest pain as a secondary contact cause were excluded, as were chest pain patients with dyspnea as a secondary contact cause. Such overlap was present in only 147 (5%) of the patients.

The date of death was obtained from the Swedish National Population Registry longitudinally up to 31 December 2015. Data on previous medical conditions were retrieved as all the International Classification of Diseases 10th Revision (ICD-10) diagnoses made within the region (region Skåne) in the five years preceding the ED presentation.

### 2.5. Statistical Analyses

Patient characteristics, comorbidities, and outcomes were compared between the dyspnea and chest pain groups using *t*-tests for continuous variables and chi-square tests for categorical variables. Differences in outcomes were analyzed using linear regression for continuous outcomes and logistic regression for categorical outcomes. Time of death was analyzed using Cox regression. Associations were expressed with 95% confidence intervals (CI) and were estimated unadjusted and adjusted for potential confounders: age, sex, centre, CCI, CRP, hs-cTnT, and arrival by ambulance. Statistical significance was defined as a two-sided *p* value <0.05. Non-normally distributed continuous variables were analyzed using Wilcoxson's rank sum test and were reported as median (IQR). Statistical analyses were conducted using the software packages Stata, version 14.2 (StataCorp LP; College Station, TX) and SAS, version 9.3 (SAS Institute, Inc., Cary, NC).

## 3. Results

We included a total of 29,291 patients (mean age 58.3 years; 49% women) who presented to the ED of Helsingborg (51%) or Lund (49%) with a primary or secondary complaint of dyspnea (*n* = 8,812) or chest pain (*n* = 20,479). Characteristics for the groups are shown in Table 1. Compared with chest pain patients, dyspnea patients were older, more often female and had more comorbidity in the form of COPD, heart failure, pulmonary embolism, and pneumonia. However, there was little difference in previous coronary artery disease. The most common previous diseases in the dyspnea group were COPD, heart failure, asthma, and pneumonia, whereas, among those with the chest pain, they were angina pectoris and acute myocardial infarction (AMI). Average CRP and hs-cTnT levels were higher in patients with dyspnea than with chest pain.

The article "Outcomes in Emergency Department Patients with Dyspnea versus Chest Pain: A Retrospective Consecutive Cohort Study" was published in 2022. Journal: Emerg Med Int.

Seasonal and diurnal variations in the ED presentation for each contact cause are shown in Figures 1(a) and 1(b). Dyspnea patients had a distinct “peak” in the winter to early spring of the year, while patients with chest pain presented to the ED more evenly throughout the year. Diurnal presentation patterns were similar in the two groups.

Outcomes are shown in Table 2. Compared to chest pain patients, dyspnea patients were more often admitted to in-hospital care (47.9% *vs.* 29.5%), including to the ICU (1.4% *vs.* 0.1%), and had longer hospital stays and more ED revisits. Mortality was assessed during a median of 3.5 years (range 0–6.0 years), yielding a total of 97,812 person-years of follow-up. Mortality was clearly higher in dyspnea patients at all points of follow-up. As shown in Figure 2, cumulative mortality over time was markedly higher in dyspnea patients (2,917 deaths; incidence rate 0.12 (95% CI, 0.11–0.12) per person-year) compared with chest pain (1,612 deaths; incidence rate 0.022 (95% CI, 0.021–0.023) per person-year). In a Cox regression analysis of time from ED visits to death, dyspnea was associated with five-fold increased mortality compared to chest pain, crude HR 5.1 (95% CI, 4.8–5.4). When controlling for centre and markers of disease severity (age, sex, CCI, CRP, Hs-cTnT, and arrival by ambulance), dyspnea was associated with a two-fold higher mortality, adjusted HR 2.2 (95% CI, 2.0–2.4; *p* < 0.001).

## 4. Discussion

In this large consecutive cohort of ED patients, the main findings were that dyspnea patients had a markedly higher rate of hospitalization, an almost ten-fold higher ICU admittance, more ED revisits, and a five to ten times higher crude mortality compared with ED patients with chest pain. The excess risks in dyspnea patients decreased after adjusting for differences in disease severity (age, sex, centre, CCI, CRP, Hs-cTnT, and arrival by ambulance), indicating that the worse outcomes were largely attributed to more severe underlying illness.

Our study adds novel and important data on morbidity in unselected ED patients with a contact cause of dyspnea or chest pain. Dyspnea patients commonly had previous diagnoses of COPD, heart failure, asthma, and pneumonia, while angina pectoris and previous AMI were more common in chest pain patients. Diabetes and hypertension were common in both groups. Previous COPD, heart failure, asthma, and pneumonia are common in ED patients with dyspnea and have previously been reported in Europe [19], Southeast Asia, and Oceania [1]. However, our dyspnea patients less often had previous COPD or asthma compared to other studies [1, 19]. This might to some extent be explained by lifestyle factors but that needs to be investigated further. In our chest pain patients, the rate of previous angina pectoris and AMI was in accordance with previous reports [20–22].

The article "Outcomes in Emergency Department Patients with Dyspnea versus Chest Pain: A Retrospective Consecutive Cohort Study" was published in 2022. Journal: Emerg Med Int.

Dyspnea as a cause of contact was more common in the winter months compared to chest pain. A previous study suggests that ED dyspnea patients in the winter months are typically older and often have a lower respiratory tract infection, COPD, and/or heart failure [23].

Dyspnea patients had markedly worse outcomes than chest pain patients, with e.g. a 10-fold higher 7-day crude mortality, which is well in-line with previous findings of 10 times higher in-hospital mortality for dyspnea compared to chest pain patients [3]. The long-term mortality (median follow-up of 3.5 years) in our dyspnea patients was also markedly higher with a crude HR of 5.1 and an HR of 2.2 when adjusted for disease severity. This mortality estimate is similar to the HR of 1.9–2.9 reported in a comparison of dyspnea and chest pain patients after cardiac stress testing [14].

The novel finding that the HR for mortality decreased from 5.1 to 2.2 when adjusted for age, sex, centre, CCI, CRP, Hs-cTnT, and arrival by ambulance supports that the worse outcomes in the dyspnea group is partly related to more severe underlying illness. The remaining two-fold increased mortality suggests that dyspnea in itself is an independent risk factor, but other factors such as other underlying conditions, lung function and smoking [13], hypercapnia, and/or increased blood levels of creatinine, or markers of heart failure [24] could also explain the poorer outcome. In our study, 16.2% of the dyspnea patients had previous heart failure vs. 4.7% of the chest pain patients and 4.6% vs. 1.6% had renal disease. A similar pattern of worse outcomes in older patients with comorbidities of heart failure, diabetes, and renal disease has also been shown in STEMI patients presenting with dyspnea or other atypical symptoms rather than chest pain [25]. Further research to clarify the factors and mechanisms behind the bad outcome in dyspnea patients is warranted.

The article "Outcomes in Emergency Department Patients with Dyspnea versus Chest Pain: A Retrospective Consecutive Cohort Study" was published in 2022. Journal: Emerg Med Int.

A strength of this study was the large consecutive ED patient cohort with a complete follow-up of outcomes using cross-linked registry data. Several clinically relevant variables could be analyzed to evaluate the difference in outcomes between the groups. Another strength was the possibility to rinse for overlap between the two causes of contact. Overlap between the groups of dyspnea and chest pain was present in about 5% of patients, which is in line with previous studies comparing symptoms as causes of contact [24, 26]. However, in studies of individual diagnoses such as STEMI, both chest pain and dyspnea may present in up to 60% of the patients [25]. Avoiding overlap does not abolish the subjectivity of symptom categorization but is important since the chief complaint predicts outcomes and influences ED patient management before the diagnosis is known [3]. One limitation of the study was the lack of data on vital parameters and acuity scores at ED triage, preventing analysis related to severity of illness on arrival. Data were also unavailable on underlying factors such as smoking habits, blood tests, including B-type natriuretic peptides, or data on heart and lung functions. As mentioned, these variables and different markers of disease severity may be relevant to further explain the differences in outcomes between the groups.

The increased morbidity and mortality of dyspnea patients in this study strengthen the evidence that a chief complaint of dyspnea in itself is an early marker of severe disease, indicating a need for prioritized care. The finding that morbidity and mortality to a large part were explained by underlying factors indicates that it should be possible to create risk-stratification tools for ED dyspnea patients, quickly identifying those who will benefit from specific and/or aggressive care, ICU admission, close follow-up at discharge, or perhaps a more palliative approach.

## 5. Conclusions

This large consecutive cohort study indicates that compared with chest pain patients, ED dyspnea patients are older and have more comorbidity and that they fare markedly worse in terms of hospitalization and mortality. Our findings support that a contact cause of dyspnea is a marker of severe illness and should warrant fast diagnostics and treatment to lower the risk of a bad outcome.

## Figures and Tables

**Figure 1:** (a) ED visits by month of the year. (b) ED visits by time of the day.

**Figure 2:** Mortality after ED contact for dyspnea vs. chest pain.

**Table 1:** Patients characteristics.

	Dyspnea	Chest pain	*P* value
Number of patients	8,812	20,479	
Men	3,994 (45.3%)	10,962 (53.5%)	<0.001
Age, mean (SD)	64.2 (20.7)	55.7 (18.7)	<0.001
Previous or coexisting disease			
Charlson comorbidity index, median (IQR)	1 (0, 2)	0 (0, 1)	<0.001
Angina pectoris	731 (8.3%)	1,940 (9.5%)	0.001
Acute myocardial infarction	737 (8.4%)	1,572 (7.7%)	0.045
Heart failure	1,427 (16.2%)	967 (4.7%)	<0.001
Cardiac arrhythmia	365 (4.1%)	693 (3.4%)	0.001
Valvular heart disease	295 (3.3%)	322 (1.6%)	<0.001
Pulmonary artery disease	493 (5.6%)	616 (3.0%)	<0.001
Pulmonary embolism	227 (2.6%)	153 (0.7%)	<0.001
Cerebrovascular disease	721 (8.2%)	849 (4.1%)	<0.001
Hypertension	2,999 (34.0%)	5,134 (25.1%)	<0.001
Chronic obstructive pulmonary disease	1,489 (16.9%)	735 (3.6%)	<0.001
Asthma	1,117 (12.7%)	1,167 (5.7%)	<0.001
Respiratory insufficiency	267 (3.0%)	162 (0.8%)	<0.001
Hypoventilation	13 (0.1%)	7 (<1%)	<0.001
Pulmonary fibrosis	92 (1.0%)	36 (0.2%)	<0.001
Pneumonia	814 (9.2%)	511 (2.5%)	<0.001
Bronchitis	141 (1.6%)	141 (0.7%)	<0.001
Tuberculosis	10 (0.1%)	10 (<0.1%)	0.052
Pneumothorax	52 (0.6%)	21 (0.1%)	<0.001
Diabetes	1,303 (14.8%)	1,931 (9.4%)	<0.001
Renal disease	408 (4.6%)	328 (1.6%)	<0.001
Anxiety disorder	650 (7.4%)	1,498 (7.3%)	0.85
Arrival by ambulance	282 (3.2%)	711 (3.5%)	0.24
High sensitivity troponin *T*, median (IQR), *n* = 22959	15.0 (4.0, 37.0)	4.5 (4.0, 11.0)	<0.001
C-reactive protein, median (IQR), *n* = 25331	11.0 (2.8, 48.0)	1.7 (0.7, 4.8)	<0.001
Hemoglobin, median (IQR), *n* = 14855	136.0 (125.0, 148.0)	143.0 (133.0, 152.0)	<0.001

Data presented as mean (standard deviation) or frequency (%) unless otherwise specified.

The article "Outcomes in Emergency Department Patients with Dyspnea versus Chest Pain: A Retrospective Consecutive Cohort Study" was published in 2022. Journal: Emerg Med Int.

**Table 2:** Outcomes in patients with dyspnea vs. chest pain.

Outcomes	Dyspnea, *N* = 8,812	Chest pain, *N* = 20,479	Unadjusted, dyspnea vs. chest pain (95% CI)	Adjusted, dyspnea vs. chest pain (95% CI)^*∗*^
Time in emergency department (hours), median (IQR)	3.8 (2.5, 5.4)	3.3 (2.3, 4.8)	0.4 (0.3–0.5)^#^	0.6 (0.5–0.7)^#^
Admitted to hospital	4,222 (47.9%)	6,040 (29.5%)	2.2 (2.1–2.3)	1.2 (1.1–1.3)
Admitted to ICU	120 (1.4%)	27 (0.1%)	10.5 (6.9–15.9)	8.16 (3.7–18.2)
Length of hospital stay among admitted (days), median (IQR)	4.00 (2.00, 7.00)	2.00 (1.00, 4.00)	2.5 (2.2–2.8)^#^	1.6 (1.3–1.9)^#^
Revisit within 7 days	368 (4.2%)	715 (3.5%)	1.2 (1.1–1.4)	1.4 (1.1–1.6)
Revisit within 30 days	967 (11.0%)	1,463 (7.1%)	1.6 (1.5–1.7)	1.5 (1.2–1.7)
Revisit within 1 year	2,837 (32.2%)	4,808 (23.5%)	1.55 (1.5–1.6)	1.1 (1.0–1.2)
Mortality within 7 days	291 (3.3%)	70 (0.3%)	10.0 (7.7–12.9)	2.9 (1.9–4.4)
Mortality within 30 days	581 (6.6%)	135 (0.7%)	10.6 (8.8–12.9)	3.4 (2.5–4.6)
Mortality within 1 year	1,599 (26.7%)	576 (5.2%)	6.6 (6.0–7.3)	1.7 (1.4–2.1)

^*∗*^Adjusted for age, sex, centre, Charlson comorbidity index, CRP, Hs-cTnT, and arrival by ambulance. Estimates are odds ratios (for binary outcomes) using logistic regression, or ^#^mean difference using linear regression (for continuous outcomes).

The article "Outcomes in Emergency Department Patients with Dyspnea versus Chest Pain: A Retrospective Consecutive Cohort Study" was published in 2022. Journal: Emerg Med Int.

## Data Availability

The datasets used and/or analyzed during this study are available from the corresponding author upon request.
